The article "Diagnosing the Stage of Hepatitis C Using Machine Learning" was published in 2021. Journal: J Healthc Eng.

# Diagnosing the Stage of Hepatitis C Using Machine Learning

**DOI:** 10.1155/2021/8062410

**Published:** 2021-12-10

**Authors:** Muhammad Bilal Butt, Majed Alfayad, Shazia Saqib, M. A. Khan, Munir Ahmad, Muhammad Adnan Khan, Nouh Sabri Elmitwally

**Affiliations:** ^1^Department of Computer Science, Lahore Garrison University, Lahore 54000, Pakistan; ^2^College of Computer and Information Sciences, Jouf University, Sakaka 72341, Saudi Arabia; ^3^Riphah School of Computing & Innovation, Faculty of Computing, Riphah International University, Lahore Campus, Lahore 54000, Pakistan; ^4^School of Computer Science, National College of Business Administration & Economics, Lahore 54000, Pakistan; ^5^Department of Software, Gachon University, Seongnam, Gyeonggi-do 13557, Republic of Korea; ^6^Department of Computer Science, Faculty of Computers and Artificial Intelligence, Cairo University, Giza 12613, Egypt; ^7^School of Computing and Digital Technology, Birmingham City University, Birmingham B4 7XG, UK

## Abstract

Hepatitis C is a prevalent disease in the world. Around 3 to 4 million new cases of Hepatitis C are reported every year across the globe. Effective, timely prediction of the disease can help people know about their Stage of Hepatitis C. To identify the Stage of disease, various noninvasive serum biochemical markers and clinical information of the patients have been used. Machine learning techniques have been an effective alternative tool for determining the Stage of this chronic disease of the liver to prevent biopsy side effects. In this study, an Intelligent Hepatitis C Stage Diagnosis System (IHSDS) empowered with machine learning is presented to predict the Stage of Hepatitis C in a human using Artificial Neural Network (ANN). The dataset obtained from the UCI machine learning repository contains 29 features, out of which the 19 most reverent are selected to conduct the study; 70% of the dataset is used for training and 30% for validation purposes. The precision value is compared with the proposed IHSDS with previously presented models. The proposed IHSDS has achieved 98.89% precision during training and 94.44% precision during validation.

## 1. Introduction

Hepatitis C is a type of liver disease which is instigated due to the “Hepatitis C Virus (HCV)” [1]. It is considered to be the root of liver cancer. This virus can produce or instigate chronic Hepatitis and acute Hepatitis, ranging from mild illness of a few weeks to serious illness lasting until death [1, 2]. HCV is a sort of bloodborne virus. The common forms of infection are applied to small quantities of blood [3]. It can spread due to used drug injection, unsafe healthcare, transfusion of the blood or blood plasma, unsafe practices of injections, and sexual practices.

The HCV infection can be cured in 95% of cases by using antiviral infections, resulting in reduced death risk due to liver cancer and cirrhosis. Still, very few have access to treatment and diagnosis [2]. Most of the people having Hepatitis C do not show any symptoms immediately. Still, after the period of two weeks to six months when the HCV enters the bloodstream, the following symptoms can be noticed, which are mentioned in Table 1 [2, 3].

The first six months of the HCV infections are known as acute Hepatitis or short-term phase Hepatitis, and, after six months, it goes into the chronic phase resulting in long-term illness. The HVC attacks the liver. As a result, the immune system of the body discharges inflammatory substances. These inflammatory substances invigorate the liver to produce fibrous protein, such as collagen, to repair the damage [2, 3]. The bolster of the scar tissues in the liver is known as fibrosis. This fibrosis can prevent the flow of blood to liver cells which will change the function of the liver. Over time, the liver cells die, and the liver stops functioning normally [4].

The “METAVIR score” is the method that is used to measure fibrosis in people with HVC. Scoring is divided into five stages which are shown in Table 2 [5, 6].

AI applications in healthcare are rapidly growing with each passing day. In recent years, AI and medicine projects attracted more attention than many other projects from the world economy [7]. AI applies in medicine to the use of automated diagnostic processes and the monitoring of individuals who need healthcare [8]. Increased use of AI in prescribing medication would allow it to automate a significant amount of the process and free up time for medical experts to carry out other duties that cannot be automated [7].

Classification is an important activity in data mining and machine learning to predict potential data object classes. Data mining uses data analysis techniques to find information and relationships within data to predict validity. Machine learning algorithms capture the data and use it to create models to take intelligence-based actions. Many authors have investigated machine learning algorithms in several areas over the last few decades to construct prediction models based on clinical records, such as determining the presence of Hepatitis C in a patient based on clinical and biochemical data.

For diagnosing the Stage of Hepatitis C that will help doctors to treat the disease at an early stage and save the patient's life, different techniques like Neurofuzzy, Gaussian Naive Bayes, Decision Trees, and Support Vector Machine (SVM) were used to diagnose Hepatitis C and its Stages. In this study, the Intelligent Hepatitis C Stage Diagnoses System (IHSDS) has been presented using an Artificial Neural Network with all the advantages such as high accuracy rates of recognition, easy structure, small-sample problem-solving capability, and strong generalization. The structure of the paper is as follows: related work is presented in the second section, which is followed by the proposed system in the third section. The fourth section shows the results of the proposed IHSDS, after which the performance evaluation is done, and the conclusion is given at the end in the fifth section.

## 2. Related Work

The HCV-infected patients can be monitored by analyzing the staging of liver fibrosis in “chronic Hepatitis C” (CHC). It can be used to determine the disease's prognosis, select the optimal medication time, and predict treatment response. Although liver biopsy has also been adopted as a more accurate diagnosis approach, it still has some disadvantages, such as invasiveness, the possibility of sampling error, and the cost of monitoring. Clinical information such as age, body mass index (BMI), and gender and noninvasive methods such as blood serum markers (alanine aminotransferase (ALT), aspartate aminotransferase (AST), white blood cell (WBC) count, glucose, hemoglobin (Hb), platelet count, the quantity of HCV RNA, red blood cell (RBC) count, etc.) are used to predict the fibrosis stage. As a result, serum biomarkers and clinical data were combined to design a classification model for predicting the fibrosis stage. Various machine learning classification algorithms have been utilized in prior studies, and their accuracies are discussed here.

Tsvetkov et al. stated that the purpose of the study was to design a model based on machine learning for diagnosing the Stage of liver fibrosis in the patients. The researchers examined 1240 patient records with chronic viral Hepatitis C. Machine learning models were developed and tested using data from 689 patients grouped by Stage of liver fibrosis. Essential predictors were chosen from nine usual prognostic factors. They achieved the highest accuracy of 80.56% [9].

In the research by Akella et al., the goal of the study was to develop clinical risk models to predict the degree of fibrosis in chronic Hepatitis C patients with ML algorithms. The nine ML algorithms were built based on an Egyptian cohort dataset and depended on demographic patients and traditional serum laboratory values. One of their models (Extreme Gradient Boosting) estimated the fibrosis with 81% precision. In addition, they concluded that most of their models outperformed many existing diagnostic alternatives in this patient population to evaluate fibrosis [10].

Gawrieh aimed to propose an integrated artificial intelligence (AI) based automated model to detect and estimate fibrosis and assess the architectural pattern in nonalcoholic fatty liver disease (NAFLD) liver biopsies. The research has used digital images of liver biopsies of patients with nonalcoholic fatty liver disease (NAFLD) with varying fibrosis levels. To identify fibrosis patterns, they used a Support Vector Machine (SVM) and achieved an accuracy of 85.6% [11].

The study by Nandipati et al. aimed to develop the performance-based comparisons between multiclass and binary class labels of the same dataset, not restricted to tool comparison, and to understand which selected features play a vital role in the Hepatitis C Virus (HCV) prediction by applying a dataset of Egyptian patients. The highest precision was shown by Random Forest (54.56%, Python) and KNN (51.06%, R) in binary class and multiclass labels, respectively [12].

Barakat et al. used Random Forest, APRI, and FIB-4 to develop a model for prediction and staging of Hepatic Fibrosis in Egyptian children having Hepatitis C Virus. They achieved the highest 90.3% precision with the random forest algorithm. The other models APRI and FIB-4 obtained 78% and 74% accuracies, respectively [13].

Li et al.'s retrospective dataset, which includes 920 patients, was used to establish Random Forest Classifier (RFC), Decision Tree Classifier (DTC), Support Vector Classifier (SVC), and Logistic Regression Classifier (LRC) for assessment of liver fibrosis severity. The highest precision of 83% was achieved with the RFC model [14].

Hashem et al. used a genetic algorithm, decision tree, multilinear regression models, and particle swarm optimization to predict advanced fibrosis risk and achieved the highest precision of 84.4% [15].

### 2.1. Limitation of Related Work

All the previously presented approaches have a few of the weaknesses mentioned below:

- Low accuracy: Most of the approaches in literature [9, 11, 14] have achieved low accuracy (not even above 90% in some cases). It gets difficult for the doctors and patients to rely on these results only.
- Experiments with fewer parameters: Some of the previously presented methods [9, 11, 14] have used a fewer number of parameters. They skip a few of the important factors in the prediction of fibrosis in a liver.
- Experiments on fewer samples: It is another issue with previous approaches [11, 13] that fewer instances are used in experiments, which compromises the overall performance and accuracy of models.

Keeping the limitation of previous methods in mind, we have eliminated these deficiencies in our work. This study was conducted using a big number of parameters that play an important role in diagnosing the degree of fibrosis in a patient. Moreover, the experiments will be performed on a more significant number of instances which will untimely increase the accuracy of our model and make it more reliable. We have presented the following important contributions in this article:

- Increased the number of parameters for conducting this study.
- Performed experiments on a big number of samples.
- Increased the accuracy of the prediction of the degree of fibrosis.

## 3. The Proposed System

We have proposed a new model in this article for diagnosing the Stage of Hepatitis C using an Artificial Back-Propagation Neural Network. The complete step-by-step approach of the proposed model is shown in Figure 1.

Various sensors are continuously collecting data from the environment, and physical quantities are transformed into measurements. Different sensors are connected with the sensor board through various topologies. Each sensor node acquires a subset from collected samples for locally compacting and summing up the random signal.

The data acquisition layer is used to acquire data like symptoms of Hepatitis C from sensors and the data like age, gender, and so forth from the user for further use. Preprocessing will be performed on collected data to transform raw data into an understandable format. Data from the real world may contain errors, can be inconsistent, and often can be incomplete. In this layer, we used missing values and mean normalization for data coding, and the moving average method with a five-filter size will be used to mitigate the noisy data. The raw data is prepared using data processing for further processing.  Table 3 shows the coding technique for data transformation.

In this research, the Hepatitis C patient dataset titled “HCV-Egy-Data” is obtained from the UCI machine learning repository [16]. It includes 1385 observations, where each sample has 29 properties, out of which 19 properties are selected. The value of attribute “histological staging” in this dataset indicates the Stage of the patient. There are 336 (24.26%) cases in class 1, 332 (23.97%) cases in class 2, 355 (25.63%) cases in class 3, and 362 (26.14%) cases in class 4. All properties of the dataset are detailed in Table 3.

The proposed model predicts the Stage of Hepatitis C using the neural network with the help of a back-propagation algorithm. In the proposed IHSDS, the application layer is further divided into two sublayers: the prediction layer and the performance layer. In the prediction layer, the first 18 attributes are used as inputs to train the proposed model. The attribute named “histological stage” is the predicted output variable based on these 18 input attributes. The prediction layer further contains an input layer, a hidden layer, and an output layer. The input layer includes 18 neurons, the hidden layer contains 90 neurons, and the output layer contains one neuron. Stage of Hepatitis C is predicted using a back-propagation algorithm. The achieved results are evaluated in precision, miss rate, and mean square error in the performance layer.

It will be stored in the cloud for validation purposes and further processing if the required precision is achieved; otherwise, the weights will be updated if the required precision is not achieved. The data from the cloud is imported into the validation layer. The input data acquired from IoMT sensors and users will be fed into the model after preprocessing for testing purposes. The proposed IHSDS will predict the Stage of Hepatitis C. Finally, the patient will be recommended to the doctor if the Stage of Hepatitis C is diagnosed; otherwise, the result will be discarded.

This research work predicts the Stage of Hepatitis C by using the back-propagation algorithm of the Artificial Neural Network model. This model is used to gain the maximum precision in the prediction of the Stage of Hepatitis C with the defined structure. The model comprises an input layer, hidden layer, and output layer. The design of the neural network is composed using feedforward and back-propagation of error. In feedforward, the information from the input layer to the hidden layer is processed and transferred towards the output layer. The back-propagation error of the process is used to reduce the error if the output layer cannot accept it. The values of weights are adjusted and transferred back to feedforward.

In this study, ANN architecture is built using the back-propagation algorithm. Different stages involved in the back-propagation algorithm include reading the training data, building and connecting the ANN layers (this includes preparing weights, biases, and activation function of each layer), predicting error, updating parameters, and prediction precision. Every neuron in the hidden layer uses the activation function. We used a sigmoid activation function in this network. (1) shows the sigmoid function for input, whereas the sigmoid function for the hidden layer of proposed IHSDS is written in (2):

(1) $$\begin{array}{c} {ų}_{j}=b_{1}+\sum_{i=1}^{m}\left(h_{ij}\times \;z_{i}\right), \end{array}$$

(2) $$\begin{array}{c} \rho_{j}=\;\frac{1}{1+\;e^{-{ų}_{j}}}\;\text{where }j=\;1,2,3\ldots n. \end{array}$$

Equation (3) shows that input is taken from the output layer.

(3) $$\begin{array}{c} {ų}_{k}=b_{2}+\;\sum_{j=1}^{n}\left({ŧ}_{jk}\times \;{ƥ}_{j}\right). \end{array}$$

Equation (4) shows the activation function for the output layer.

(4) $$\begin{array}{c} {ƥ}_{k}=\;\frac{1}{1+\;e^{-{ų}_{k}}}\;\text{where}\;k=\;1,2,3\ldots z. \end{array}$$

Equation (5) shows the sum of all squared error functions to calculate the error for output neurons, where *γ*_*k*_ represents the desired output and *ρ*_*k*_ represents the predicted output.

(5) $$\begin{array}{c} E=\;\frac{1}{2}\;\sum_{k}{\left(\gamma_{k}-\rho_{k}\right)}^{2}, \end{array}$$

and the rate of change in output layers weights is shown as

(6) $$\begin{array}{c} \Delta W\propto -\;\frac{6E}{6W},\;\Delta {ŧ}_{j,k}=\;-\;\varepsilon \;\frac{6E}{{ŧ}_{j,k}}. \end{array}$$

Equation (7) is used to substitute the values; the values of updated weights can be obtained using

(7) $$\begin{array}{c} \Delta \;{ŧ}_{j,k}=\;-\;\varepsilon \;\frac{6E}{6\gamma_{k}}\;\times \;\frac{6\gamma_{k}}{6{ų}_{k}}\;\times \;\frac{6{ų}_{k}}{6{ŧ}_{j,k}}, \end{array}$$

(8) $$\begin{array}{c} \Delta \;{ŧ}_{j,k}=\;\varepsilon \left(\gamma_{k}-\rho_{k}\right)\times \rho_{k}\left(1-\rho_{k}\right)\times \left(\rho_{j}\right)\;, \end{array}$$

where

(9) $$\begin{array}{c} S_{k}=\;\left(\gamma_{k}-\;\rho_{k}\right)\;\times \rho_{k}\left(1-\rho_{k}\right),\\ \Delta h_{i,j}\propto -\;\left[\sum_{k}\frac{6E}{\;6\rho_{k}}\times \frac{\;6\rho_{k}}{6{ų}_{k}}\times \frac{6{ų}_{k}}{\;6\rho_{j}}\right]\times \frac{\;6\rho_{j}}{6{ų}_{j}}\times \frac{6{ų}_{j}}{6h_{i,j}}\;,\\ \Delta h_{i,j}\propto -\;\left[\sum_{k}\frac{6E}{\;6{ƥ}_{k}}\times \frac{\;6{ƥ}_{k}}{6{ų}_{k}}\times \frac{6{ų}_{k}}{\;6{ƥ}_{j}}\right]\times \frac{\;6\rho_{j}}{6{ų}_{j}}\times \frac{6{ų}_{j}}{6h_{i,j}}\;,\\ \Delta h_{i,j}=\;\varepsilon \;\left[\underset{k}{\sum }\left(\gamma_{k}-\;\rho_{k}\right)\times \rho_{k}\left(1-\;\rho_{k}\right)\times \left({ŧ}_{j,k}\right)\right]\times \rho_{k}\left(1-\;\rho_{k}\right)\times \chi_{i},\\ \Delta h_{i,j}=\;\varepsilon \;\left[\underset{k}{\sum }\left(\gamma_{k}-\rho_{k}\right)\times {ƥ}_{k}\left(1-\rho_{k}\right)\times \left({ŧ}_{j,k}\right)\right]\times \rho_{j}\left(1-\rho_{k}\right)\times \chi_{i},\\ \Delta h_{i,j}=\;\varepsilon \left[\underset{k}{\sum }S_{k}\left({ŧ}_{j,k}\right)\right]\times \rho_{j}\left(1-\;\rho_{j}\right)\times \chi_{i},\\ \Delta h_{i,j}=\varepsilon S_{j}\chi_{i}, \end{array}$$

where

(10) $$\begin{array}{c} S_{j}=\left[\sum S_{k}\left({ŧ}_{j,k}\right)\right]\times \rho_{j}\left(1-\rho_{j}\right), \end{array}$$

and weights and bias update between output and hidden layers are shown as

(11) $$\begin{array}{c} {ŧ}_{j,k}\;\left(t+1\right)=\;{ŧ}_{j,k}\left(t\right)+\varrho_{F}\;△{ŧ}_{j,k}. \end{array}$$

Input and hidden layer updates are shown as

(12) $$\begin{array}{c} h_{i,j}\left(t+1\right)=\;h_{i,j}\left(t\right)+\varrho_{F}\;\Delta h_{i,j}. \end{array}$$

The learning rate of artificial back-propagation neural network is *ϱ*_*F*_ and the convergence of ABPNN depends on the good careful selection of *ϱ*_*F*_.

## 4. Results and Discussion

Simulations of the results are performed using the MATLAB R2019a tool. The dataset used to perform simulations is taken from the UCI repository [16]. It contains 1385 samples, out of which 969 samples (70% of the dataset) are used for training the model, and the remaining 416 samples (30% of the dataset) are used for validation purposes. The 969 samples for training include samples from all classes (70% of each class).

A confusion matrix represents the information about actual and predicted results obtained by the classification model. The performance of the system can be evaluated with the help of this matrix. The confusion matrices for training and validation are shown in Tables 4 and 5, respectively.

Table 4 shows the proposed IHSDS prediction of the Hepatitis C Stage during the training phase. A total of 968 samples are used for training which are further divided into 235, 232, 248, and 253 samples of class Stage I, Stage II, Stage III, and Stage IV, respectively.

213 samples of Stage I class are correctly predicted, which indicates true positive; on the other hand 11, 5, and 6 samples are incorrectly predicted in Stage II, Stage III, and Stage IV, respectively, which indicates false positive.

223 samples of Stage II class are correctly predicted, which indicates true positive; on the other hand, 3, 2, and 4 samples are incorrectly predicted in Stage I, Stage III, and Stage IV, respectively, which indicates false positive.

232 samples of Stage III class are correctly predicted, which indicates true positive; on the other hand, 5, 7, and 4 samples are incorrectly predicted in Stage I, Stage II, and Stage IV, respectively, which indicates false positive.

228 samples of Stage IV class are correctly predicted, which indicates true positive; on the other hand, 9, 9, and 7 samples are incorrectly predicted in Stage I, Stage II, and Stage III, respectively, which indicates false positive.

Table 5 shows the proposed IHSDS prediction of the Hepatitis C Stage during the validation phase. A total of 417 samples are used for validation, which are further divided into 87, 102, 113, and 115 samples of class Stage I, Stage II, Stage III, and Stage–IV, respectively.

30 samples of Stage I class are correctly predicted, which indicates true positive; on the other hand, 25, 16, and 16 samples are incorrectly predicted in Stage II, Stage III, and Stage IV, respectively, which indicates false positive.

23 samples of Stage II class are correctly predicted, which indicates true positive; on the other hand, 15, 34, and 30 samples are incorrectly predicted in Stage I, Stage III, and Stage IV, respectively, which indicates false positive.

35 samples of Stage III class are correctly predicted, which indicates true positive; on the other hand, 26, 16, and 36 samples are incorrectly predicted in Stage I, Stage II, and Stage IV, respectively, which indicates false positive.

34 samples of Stage IV class are correctly predicted, which indicates true positive; on the other hand, 24, 21, and 36 samples are incorrectly predicted in Stage I, Stage II, and Stage III, respectively, which indicates false positive.

Now to evaluate the performance of the proposed model, precision, miss rate, and mean square error (MSE) are calculated. The formulas to calculate these above metrics are given in (13), (14), and (15), respectively.  Table 6 shows the precision, miss rate, and mean square error (MSE) calculated during the training and validation phases. The proposed IHSDS gives 98.89% precision and 1.11% miss rate, respectively, during the training phase and 94.44% precision and 5.56% miss rate during the validation phase, respectively.

(13) $$\begin{array}{c} \text{Percision}=\frac{p_{i}/y_{i}+p_{k}/y_{k}}{p_{i}/y_{i}+\left(\sum_{j=1}^{z}\left(p_{j},\;j\neq i\right)\;/y_{j}\right)+p_{k}/y_{k}+\left(\sum_{i=1}^{n}\left(p_{i},\;i\neq k\right)\;/y_{k}\right)}, \end{array}$$

where *i*/*j*/*k*/l = 1, 2, 3, 4,…, *z*.

(14) $$\begin{array}{c} \text{Miss Rate}=\frac{\sum_{i=1}^{z}\left(p_{i},\;i\neq k\right)/y_{k}}{\;\sum_{i=1}^{z}\left(p_{i},\;i\neq k\right)/y_{k}+p_{i}/y_{i}}, \end{array}$$

where *i*/*k*/l = 1, 2, 3, 4,…, *z*.

(15) $$\begin{array}{c} \text{MSE}=\;\frac{1}{n}\sum_{i=1}^{n}{\left(y_{i}-\;{\tilde{y}}_{i}\right)}^{2}. \end{array}$$

The proposed IHSDS model and the methods proposed by Akella and Akella [10], Gawrieh et al. [11], Li et al. [14], and also Hashem et al. [15] are compared with a measure of evaluation, precision.

The proposed IHSDS is empowered with machine learning results with 98.89% precision value during training and 94.44% precision value during validation. The validation precision value of previous methods is compared with the proposed model in Table 7. It is justified to state that the results provided by the proposed IHSDS empowered with machine learning are better than the results provided by previously proposed methods with regard to precision.

## 5. Conclusion

Before the evolution of machine learning in the medical domain, doctors needed to do various tests to diagnose the Stage of Hepatitis C in a particular patient. The patient has to undergo unnecessary tests and check-ups to identify the disease stage during the whole diagnosis process. Its cost for the patient is too high and takes a lot of his time. There should be a preliminary test to reduce unnecessary check-ups and save the time of both (doctors and patients) by notifying them about the Stage of Hepatitis C disease in a patient so that the treatment can be started as per need. Machine learning techniques and their various algorithms are helpful for the prediction of diseases and classification based on medical data. The Artificial Neural Network (ANN) machine learning algorithm is used to conduct this study. The proposed IHSDS was trained and validated using the dataset and shows 98.89% and 94.44% precision during training and validation phases, respectively. A comparative analysis of the proposed model with previous models is also presented based on precision and miss rate, which justifies that the proposed model is better than the previously available methods.

## Figures and Tables

**Figure 1:** Proposed Intelligent Hepatitis C Stage Diagnosis System (IHSDS) empowered with machine learning.

**Table 1:** Symptoms of chronic Hepatitis C.

Symptoms	
Fever	Vomiting
Fatigue	Headache
Jaundice	Bone ache
Weight loss	Epigastric pain

**Table 2:** Stage of Hepatitis C.

Stage 0	Stage 1	Stage 2	Stage 3	Stage 4
No fibrosis	Mild fibrosis exclusive of scarring walls	Mild-to-moderate fibrosis inclusive of scarring walls	Spreading of bridged scarring to various liver parts but no cirrhosis	Severe cirrhosis or scarring

**Table 3:** Detailed description of dataset.

Sr. no.	Attribute	Value range	Interpretation	Type
1	Age	32–61	Age of patient	Predictive
2	Gender	1–2	Female = 2, male = 1	Predictive
3	BMI	22–35	Weight of patient	Predictive
4	Fever	1–2	Yes = 2, no = 1	Predictive
5	Nausea	1–2	Yes = 2, no = 1	Predictive
6	Headache	1–2	Yes = 2, no = 1	Predictive
7	Fatigue	1–2	Yes = 2, no = 1	Predictive
8	Jaundice	1–2	Yes = 2, no = 1	Predictive
9	Epigastric pain	1–2	Yes = 2, no = 1	Predictive
10	WBC	2991–12101	WBC count	Predictive
11	RBC	3816422–5018451	RBC count	Predictive
12	HGB	10–15	HGB level	Predictive
13	Plat.	9303–226464	Plat. count	Predictive
14	AST	39–128	AST level (1^st^ week)	Predictive
15	ALT 1	39–128	ALT level (1^st^ week)	Predictive
16	ALT 4	39–128	ALT level (4^th^ week)	Predictive
17	RNA 1	11–1201086	RNA count (1^st^ week)	Predictive
18	RNA 4	5–1201715	RNA count (4^th^ week)	Predictive
19	Histological staging	1–4	Stage	Class

**Table 4:** Confusion matrix for the proposed IHSDS during training.

Proposed IHSDS model (70% of the dataset in training)				
*N* = 968 (no. of samples)		Predicted output (Ƥ0, Ƥ1, Ƥ2, Ƥ3)		
Actual output (*ƴ*0, *ƴ1*, *ƴ*2, *ƴ*3)	Ƥ0 (Stage I)	Ƥ1 (Stage II)	Ƥ2 (Stage III)	Ƥ3 (Stage IV)
Input				
*ƴ*0 = 235 (Stage I)	159	28	15	16
*ƴ*1 = 232 (Stage II)	29	182	17	21
*ƴ*2 = 248 (Stage III)	19	13	200	16
*ƴ*3 = 253 (Stage IV)	17	18	25	193

**Table 5:** Confusion matrix for the proposed IHSDS during validation.

Proposed IHSDS model (30% of the dataset in validation)				
*N* = 417 (no. of samples)		Predicted output (Ƥ0, Ƥ1, Ƥ2, Ƥ3)		
Actual output (*ƴ*0, *ƴ*1, *ƴ*2, *ƴ*3)	Ƥ0 (Stage I)	Ƥ1 (Stage II)	Ƥ2 (Stage III)	Ƥ3 (Stage IV)
Input				
*ƴ*0 = 87 (Stage I)	30	25	16	16
*ƴ*1 = 102 (Stage II)	15	23	34	30
*ƴ*2 = 113 (Stage III)	26	16	35	36
*ƴ*3 = 115 (Stage IV)	24	21	36	34

**Table 6:** Performance evaluation of the proposed IHSDS during training and validation.

		Samples [#]	Precision (%)	Miss rate (%)	MSE (%)
Proposed IHSDS	Training	969	98.89	1.11	3.63917 × 10^−3^
	Validation	416	94.44	5.56	3.22580 × 10^−2^

**Table 7:** Comparison of the proposed model with previously presented models using validation precision.

Literature	Dataset description	Precision (%)	Miss rate (%)
Extreme Gradient Boosting [10]	HCV Egyptian cohort dataset (1385 samples of 6 features are used)	81.00	19.00
Random Forest [14]	HCV dataset by Clinical Research Committee of Second Xiangya Hospital, Central South University (920 samples of 9 features are used)	83.00	17.00
Support Vector Machine (SVM) with linear kernel [11]	18 liver biopsy images of the trichrome (TC) stained slides	85.60	14.40
Random Forest [13]	Dataset of children attending hospital outpatient clinic (166 samples of 14 features are used)	90.30	9.70
Proposed IHSDS	HCV Egyptian cohort dataset (1385 samples of 18 features are used)	94.44	5.56

## Data Availability

The simulation data used in this study to support the findings are available upon request from the corresponding author.
